This article has been retracted.

# Ropivacaine and Lidocaine in Double Eyelid Blepharoplasty: A Comparative Analysis

**DOI:** 10.1155/2022/7029570

**Published:** 2022-05-29

**Authors:** Shaobo Liu, Zheng Chu

**Affiliations:** ^1^Department of Plastic Surgery, Pangang Group General Hospital, Panzhihua, Sichuan, China; ^2^Department of Cosmetic Surgery, Xinjiang Plastic Surgery Hospital, Urumqi, China

## Abstract

Double eyelid blepharoplasty is an operation of changing the structure of the eyelid and reshaping the eyelid to form a new upper eyelid fold. This prospective randomized controlled study aimed to compare and evaluate the effect of ropivacaine and lidocaine in double eyelid blepharoplasty. A total of 120 patients who underwent double eyelid blepharoplasty in the beauty department of our hospital from January 2019 to July 2021 were enrolled and randomized (1 : 1) into the control group (1% lidocaine-epinephrine mixture) and the study group (0.75% ropivacaine-epinephrine mixture) via the random number table method. The 0.75% ropivacaine-epinephrine mixture led to lower Wong-Baker FACES Pain Rating visual analog scale score from 2 h to 1 d after surgery versus 1% lidocaine-epinephrine mixture (all *P* < 0.05). The operation time, intraoperative anesthetic drug dosage, and intraoperative blood loss were similar in the two groups (all *P* < 0.05). The 0.75% ropivacaine-epinephrine mixture resulted in a lower postoperative swelling score, but a higher patient satisfaction score versus 1% lidocaine-epinephrine mixture (all *P* < 0.05). The safety profiles of the two groups were similar (all *P* < 0.05). Both lidocaine and ropivacaine produce desirable anesthesia effects in double eyelid blepharoplasty. Ropivacaine can significantly reduce postoperative pain and mitigate postoperative swelling, with better satisfaction, and is thus worthy of further promotion.

## 1. Introduction

Double eyelid blepharoplasty is an operation of changing the structure of the eyelid and reshaping the eyelid to form a new upper eyelid fold [1, 2]. Aesthetically, double eyelids are more three-dimensional than single eyelids, due to its wide and long clefts, rich layers, and more exposed parts of the cornea. Appropriately 40% population are single eyelid in China, and it hugely stimulates the demand for double blepharoplasty [3]. The double eyelid blepharoplasty is to alter the distribution of the original bloated eyelid tissue and establish a direct connection between the skin-orbicularis oculi muscle and the meibomian-levator aponeurosis [4, 5].

Currently, blepharoplasty mainly constitutes buried suture methods for the double eyelid blepharoplasty and incision method. The former technique sutures the meibomian-levator aponeurosis with the skin-orbicularis oculi muscle by burying sutures, forming a temporary suture fixation. However, the tissue cells of the eyelid would develop an inflammatory response to the buried suture and produce autologous collagen fibers to wrap the suture to form a replacement for autologous tissue. Worse yet is that the suture would loosen, and subsequently, the newly formed collagen fibers would replace the buried sutures [6]. The latter technique is performed by cutting the skin horizontally along the designed incision line, readjusting the volume of orbital septum fat, thinning the orbicularis oculi muscle, and adjusting the binding status of the levator aponeurosis and the tarsal plate to form the direct connection between the skin-orbicularis oculi muscle and the meibomian-levator aponeurosis [7].

Due to the merits of the long-lasting effect and wide-range indications, the incision method has been extensively recognized. However, double eyelid blepharoplasty is highly demanding regarding intraoperative local infiltration anesthesia and postoperative analgesia [8]. Excellent anesthesia and analgesia can reduce tension, anxiety, and fear caused by pain and contribute to good surgical results and satisfaction. Lidocaine is a commonly used drug in anesthesia for double eyelid incision, whereas it has shortcomings such as short action time and skin swelling [9]. Ropivacaine is a L-body long-acting amide local anesthetic. It can reversibly block impulse conduction along nerve fibers by blocking the flow of sodium ions into the cell membrane of nerve fibers; moreover, it has dual effects of anesthesia and analgesia and therefore is prevalent in the surgical area block and epidural anesthesia and postoperative epidural [10]. As previously noted, lidocaine is a medium effect local anesthetic and the ropivacaine is a long-term local anesthetic. Both are used in surgery, and their differences have yet been studied to date. To address this gap, we intended to compare the efficacy of the two anesthetic methods.

## 2. Materials and Methods

### 2.1. Baseline Information

This study is a prospective randomized controlled study, using a double-blind method. A total of 120 subjects who underwent double eyelid blepharoplasty in the beauty department of our hospital from January 2019 to July 2021 were enrolled. This study followed the ethical principles proposed in the Declaration of Helsinki [11] and was reviewed by the Ethics Committee of Xinjiang Plastic Surgery Hospital, no. Hps13/307. All subjects were informed of surgical risks and expected surgical results before enrollment and were informed of the research protocol and provided the signed consent form.

### 2.2. Inclusion and Exclusion Criteria

#### 2.2.1. Inclusion Criteria

The inclusion criteria were as follows: both sides were single eyelid; aged 18–35 years; American Society of Anesthesiologists (ASA) [12] grades I-II; visual, lacrimal gland, and eyelid functions were normal; and signed an informed consent form voluntarily.

#### 2.2.2. Exclusion Criteria

The exclusion criteria were as follows: drooping eyelids, history of eye surgery, or previous double eyelid surgery; weak muscle strength of the eyelid levator muscle or other neuromuscular system or congenital diseases; eye trauma, varus or valgus, uveitis, glaucoma, fundus ophthalmopathy, and other eye diseases; allergic to lidocaine or ropivacaine; with severe hypertension, diabetes, heart, lung, renal insufficiency, and thyroid diseases; and with ocular trauma, varus or valgus, uveitis, glaucoma, fundus eye disease, and other eye diseases.

### 2.3. Surgical Methods

An upper incision was made along the lower edge of the eyebrow. The lower incision was determined based on the skin range to be removed. The skin and subcutaneous tissue were then removed. The orbicularis oculi muscle (OOM) was separated, and the OOM flap was stripped to 15 mm wide. The OOM flap was lifted, and three horizontal 3–0 nylon sutures were fixed to the periosteum, which was then covered with the superior orbital margin musculocutaneous flap. The sternal upper eyelid skin and orbital fat were removed by the eyelid crease method, and the double eyelid was adjusted and reconstructed.

### 2.4. Methods of Anesthesia

To ensure double-blindness, both the surgeon and the patient were unaware of anesthetic drugs injected. The anesthesia solution was prepared by a designated nurse. 2% lidocaine hydrochloride injection (manufacturer: Shanxi Jinxin Shuanghe Pharmaceutical Co., Ltd., batch number: H11022295) 10 ml, 0.9% normal saline 10 ml, and 1 : 1000 epinephrine 0.1 mL were mixed to prepare solution A (control group). 0.75% ropivacaine hydrochloride injection (manufacturer: Shandong Qilu Pharmaceutical Co., Ltd., batch number: H20052716) 10 ml, 0.9% normal saline 10 mL, and 1 : 0.1 mL of 1000 adrenaline were mixed to prepare solution B (study group). Anesthetic drugs were injected with a 5 mL syringe and a 26-gauge needle. The needle was gradually inserted from the outside of one eyelid for anesthesia. The dose of the drug injected on each side was about 2.0–2.5 mL. The anesthetic dose was supplemented based on the intraoperative anesthesia effect, and the intraoperative drug consumption was recorded. The operations were performed by the same surgeon. After operation, the wound was cleaned and cold-compressed with ice pack for 15 minutes; the patient was instructed to change dressing regularly and pay attention to eye hygiene.

### 2.5. Observation Indicators

#### 2.5.1. Pain Score

Wong-Baker FACES Pain Rating visual analog scale [13] was used to evaluate the pain of patients immediately after surgery, and the scores of 0–10 points indicated from painless to intolerable severe pain (Figure 1). After the patient was familiar with the scale, the pain sensation number was reported. The evaluation time includes immediately after surgery (T0), 2 h after surgery (T1), 6 h after surgery (T2), 10 h after surgery (T3), 1 d after surgery (T4), and 2 d after surgery (T5).

#### 2.5.2. Intraoperative Blood Loss and Postoperative Swelling Score

Intraoperative blood loss was evaluated by the surgeon based on the amount of blood stained by the gauze at the end of the operation, of which none was counted as 0 point, 0–5 mL as 1 point, 5–10 mL as 2 points, 10–20 mL as 3 points, and >20 mL as 4 points. The swelling was checked and evaluated when changing the dressing 1 day after operation. 1 point indicates no swelling, 2 points slight swelling, 3 points obvious swelling, 4 points difficult to open, and 5 points cannot open eyes.

#### 2.5.3. Postoperative Complications

The patient's sutures were removed 7 days after surgery, and current complications including hematoma, infection, swelling, and ecchymosis were recorded; the subjects were followed-up for 3 months after surgery to record long-term complications such as scar hyperplasia, over-shallow double eyelid, and asymmetry bilateral double eyelid.

#### 2.5.4. Subjects Satisfaction

3 months after surgery, a questionnaire survey was used to evaluate satisfaction with respect to the double eyelid effect, recovery time, and postoperative pain. Each item was scored from 1 to 4 points, indicating, respectively, dissatisfied, basically satisfied, satisfied, and very satisfied.

### 2.6. Statistical Analysis

SPSS 23.0 was employed for statistical analysis and GraphPad Prism 8.0 for graphic plotting. The measurement data are expressed as (*x* ± *s*), and the paired *t*-test was used for comparison at different time points within the group, and the two independent sample *t*-test was used for the comparison between groups. Count data and grade data are expressed as rate and examined by the chi-square test. *α* = 0.05 indicated a statistical significance.

## 3. Results

### 3.1. Patients Profile

As given in Table 1, the two groups of patients were balanced in terms of age, weight, gender, injection order, and ASA classification (all *P* < 0.05).

### 3.2. Postoperative Pain

As shown in Figure 2, the Wong-Baker scores of the two groups were lower at T0 (*P* < 0.05); from T2 to T5, the Wong-Baker scores of the study group were significantly lower than those of the control group (all *P* < 0.05); at T1 and T2, the Wong-Baker scores of the two groups were higher compared to T0 (*P* < 0.05); at T3 and T4, the Wong-Baker scores of the two groups of patients decreased significantly (all *P* < 0.05); at T5, the Wong-Baker scores of the two groups of patients were lower than those at T0 (all *P* < 0.05). No significant difference was found at all time points between the groups (*P* < 0.05).

### 3.3. Operation Time and Intraoperative Anesthetic Dose

The operation time in the control group was 35.68 ± 9.23 min, and the intraoperative anesthetic dose was 2.62 ± 0.51 mL; these in the study group were 37.16 ± 8.14 min and 2.45 ± 0.46 mL, respectively (all *P* < 0.05).

### 3.4. Intraoperative Blood Loss and Swelling Scores

As shown in Figure 3, the postoperative bleeding score of the control group was 2.59 ± 0.42 points, which was not considerably different from 2.72 ± 0.62 points of the study group (*P*=0.181); the difference in postoperative swelling score in the two groups was significant (3.15 ± 0.65 vs. 2.64 ± 0.68) (*P* < 0.001).

### 3.5. Short-Term Complications

As given in Table 2, there were 2 cases of hematoma, 1 case of infection, and 3 cases of swelling in the control group at 7 days postoperatively, while the study group had 1 case of hematoma and 1 case of infection at 7 days postoperatively. Overall, the incidence of short-term adverse reaction in the study group was similar to that in the control group (11.67% (7/60) vs. 8.33% (5/60)) (*P* > 0.05).

### 3.6. Long-Term Complications

As given in Table 3, the control group had 1 case of scar hyperplasia, 6 cases of double eyelid hyperplasia, and 3 cases of bilateral double eyelid asymmetry; the study group had 2 cases of scar hyperplasia, 1 case of shallow eyelid, and 1 case of bilateral double eyelid asymmetry. The total incidence of long-term adverse reaction in the two groups was similar (16.67% (10/60) vs. 6.67% (4/60)) (*P* > 0.05).

### 3.7. Patient Satisfaction

As given in Table 4, 0.75% ropivacaine hydrochloride injection was associated with higher total satisfaction versus 2% lidocaine hydrochloride injection (76.67% (46/60) vs. 91.67% (55/60)) (*P*=0.024). Typical cases of postoperative recovery are shown in Figure 4.

## 4. Discussion

In this study, the promising results of incision method for double eyelid blepharoplasty has been confirmed due to its deeper folds, stable postoperative double eyelid, and longer maintenance time [14]. In addition, the incision method is practical in reconstruction of the upper eyelid, eyelashes inversion, orbital septum relaxation, and upper eyelid skin relaxation [15]. However, the local anesthesia requested in the incision method raises the risk of postoperative eyelid swelling, incision infection, and scarring. Additionally, postoperative pain would hinder the recovery and thus lead to an inferior outcome. Furthermore, the participants are vulnerable to the damage in blood vessels, nerve endings, muscles, and other tissues within the incision area during the operation and even serious complications such as hematoma and ptosis. Nevertheless, there is a possibility of unsuccessful folding due to insufficient connection between the dermis and the underlying structure as a result of the improper anesthesia method, and poor intraoperative cooperation, intraoperative bleeding, postoperative pain, and swelling inevitably compromise the surgery outcome [16]. Armed with the knowledge, it is particularly imperative to choose the appropriate anesthesia method.

In the present study, ropivacaine outweighed lidocaine in terms of postoperative pain, postoperative swelling, and patient satisfaction. In clinical practice, the pros and cons of a anesthetics are measured from dimensions of the onset time, anesthesia time, and toxicity In spite of the similar property of lidocaine and ropivacaine, their pharmacokinetics and other features are varying. Nondissociated drugs are the main form of drugs passing through cell membranes, and their proportion is subjected to the drug's own dissociation constant (pKa) [17]. Lidocaine and ropivacaine are both weakly alkaline, and their pKa is 7.8 and 8.2, respectively. In the extracellular fluid, there are more nondissociated lidocaine molecules than nondissociated ropivacaine at the same concentration, which result in a better onset time of ropivacaine compared to lidocaine. In addition, ropivacaine is more fat-soluble and maintains a higher drug concentration in the cell, thereby displaying a better analgesic effect. The plasma protein binding rate of lidocaine is about 50–60%, while ropivacaine is only 6%, indicating that ropivacaine acts longer [18]. In double blepharoplasty, excessive injection of anesthetics is associated with the original anatomical structure and the outcome of the operation. Prior studies suggested that lidocaine injection is prone to cause skin swelling, itching, and bruises [19]. Ropivacaine is a new type of pure L-body long-acting amide local anesthetic, and the high doses are practical in surgical anesthesia, while the small doses are effective in sensory block and analgesia (restricted to limited nonprogressive motor nerve block). Ropivacaine can block the flow of sodium ions in the human nerve fiber cell membrane along the impulse conduction along the nerve fiber to produce a reversible block, thereby relieving the pain [20]. This interpretation is supported by the fact that the study group patients experience milder postoperative pain compared to the control group patients in the present study.

## 5. Conclusion

Both lidocaine and ropivacaine are effective anesthesia approaches in double blepharoplasty, whereas ropivacaine exhibited superior performance in reducing postoperative pain, relieving postoperative swelling, and boosting satisfaction. It merits widespread promotion.

## Figures and Tables

**Figure 1:** Schematic diagram of Wong-Baker scoring.

**Figure 2:** Comparison of postoperative pain between the two groups of patients. ^*∗∗*^*P* < 0.01. ^*∗∗∗*^*P* < 0.001.

**Figure 3:** Comparison of bleeding volume score (a) and swelling score (b) between the two groups. ^*∗∗∗*^*P* < 0.001.

**Figure 4:** Typical cases of postoperative recovery.

**Table 1:** Comparison of general information of the two groups of patients.

	Control group (*n* = 60)	Study group (*n* = 60)	*t*/*χ*^2^	*P*
Age ($\bar{x}\pm s$, years old)	29.22 ± 5.26	31.45 ± 5.64	1.195	0.234

Weight ($\bar{x}\pm s$, kg)	61.58 ± 8.24	58.19 ± 7.96	2.157	0.033

Gender			0.976	0.323
Male	16	21		
Female	44	39		

First injection site			0.835	0.361
Left	26	31		
Right	34	29		

ASA grade			0.289	0.591
I	53	51		
II	7	9		

**Table 2:** Comparison of current complications between the two groups (*n*, %).

	Hematoma	Infection	Swelling	Ecchymosis	Total rate
Control group (*n* = 60)	2	1	3	0	11.67% (7/60)
Study group (*n* = 60)	1	1	2	1	8.33% (5/60)
*χ* ^2^					0.370
*P*					0.543

**Table 3:** Comparison of long-term complications between the two groups (*n*, %).

	Scar hypertrophy	Shallow double eyelid	Symmetrical double side eyelid	Total rate
Control group (*n* = 60)	1	6	3	16.67% (10/60)
Study group (*n* = 60)	2	1	1	6.67% (4/60)
*χ* ^2^				2.911
*P*				0.088

**Table 4:** Comparison of patient satisfaction between the two groups (*n*, %).

	Very satisfied	Satisfied	Dissatisfied	Total satisfaction
Control group (*n* = 60)	21	25	14	76.67% (46/60)
Study group (*n* = 60)	28	27	5	91.67% (55/60)
*χ* ^2^				5.065
*P*				0.024

## Data Availability

No data were used to support this study.
